# Pathogenicity of local and exotic entomopathogenic fungi isolates against different life stages of red palm weevil (*Rhynchophorus ferrugineus*)

**DOI:** 10.1371/journal.pone.0255029

**Published:** 2021-07-23

**Authors:** Koko Dwi Sutanto, Mureed Husain, Khawaja Ghulam Rasool, Wahidah Hazza Al-Qahtani, Abdulrahman Saad Aldawood

**Affiliations:** 1 Plant Protection Department, College of Food and Agriculture Sciences, King Saud University, Riyadh, Saudi Arabia; 2 Department of Food Science and Nutrition, College of Food and Agriculture Sciences, King Saud University, Riyadh, Saudi Arabia; Harran Üniversitesi: Harran Universitesi, TURKEY

## Abstract

Entomopathogenic fungi are regarded as effective biocontrol agents in pest management. Different fungi isolates exhibit varying degree of pathogenicity against red palm weevil [*Rhynchophorus ferrugineus* (Olivier)]. The pathogenicity of four native isolate from Saudi Arabia (three *Beauveria bassiana* named as BbSA-1, BbSA-2, BbSA-3 and one *Metarhizium anisopliae* regarded as MaSA-1) and three exotic isolates from Indonesia (*B*. *bassiana* coded as BbIDN-1 and *M*. *anisopliae* named as MaIDN-1 and MaIDN-2) was evaluated against red palm weevil under laboratory conditions. The isolates were applied to eggs (1 day old), larvae (3 and 35 days old), pupae (5 days old) and adults (10 days old). The average mortality rate of eggs and hatched larvae was 100% in all of the isolates except BbSA-2 and BbIDN-1, where mortality was 93.3 and 90%, respectively. The lowest mortality rate (73.3%) was recorded for BbSA-3 against 3-days-old larvae; however, all other isolates caused >80% larval mortality. Meanwhile, 93.3% mortality of 35-day-old larvae was noted for MaSA-1 isolate. The highest pupa mortality (80%) was observed for MaSA-1, while remaining isolates caused >60% mortality. The isolates BbSA-1 and MaSA-1 caused 61 and 74.3% mortality in adults, respectively. The tested fungi isolates exhibited high virulence against all life stages of red palm weevil. Local isolates had higher pathogenicity than exotic isolates. The findings of the current study suggest that entomopathogenic fungi could be used as biological control agents for the management of red palm weevil. However, field studies are needed to reach the sound conclusions and practical applications.

## Introduction

Red palm weevil [*Rhynchophorus ferrugineus* (Olivier)] is one of the notorious pests in date palm orchards around the world. The larval stage of red palm weevil (RPW hereafter) is the most dangerous, which damages the trunks of date palm trees [1]. Numerous strategies have been used to manage RPW infestation, including insecticides [2, 3], pheromone traps [4–6] and microbial control agents such as nematodes [7–9], bacteria [10, 11], viruses [12, 13] and fungi [14–18]. A few of these exhibited promising response to combat RPW under field conditions [19].

Several studies have reported that microbial control agents suppressed RPW populations. For example, entomopathogenic nematodes belonging to *Steinernema* and *Heterorhabditis* genera caused 100% mortality in larvae and adults of RPW under laboratory conditions, while larval mortality was 67% under field conditions [7]. The *Bacillus spp*. reduced egg hatchability by 26.6% and caused 100% mortality of RPW [10]. Entomopathogenic virus nuclear polyhedrovirus caused 100% mortality of RPW larvae within 10 days [12]. In another study, *Beauveria bassiana* and *Metarhizium anisopliae* caused 80–82% mortality of eggs and larvae, while caused 100% mortality in adults within 2–3 weeks [14]. Similarly *B*. *bassiana* and *M*. *anisopliae* caused 95% mortality in RPW adults through an auto-contamination trap under laboratory conditions [18]. Another recent study found that different *B*. *bassiana* isolates at 3×10^8^ concentration caused 75–90% mortality after 7 days’ application when tested on third instar RPW larvae [20]. Although several studies have reported that potential of natural biocontrol agents as biocontrol agents to suppress pest populations [21–24], investigations of the pathogenicity of several fungi isolates need to be confirmed under laboratory conditions. The current study evaluated the pathogenicity of several native and exotic fungi isolates against different life stages of RPW to obtain potential isolates suitable for field applications. The results of the study will lay a strong foundation for biological control program for RPW. It was hypothesized that native isolates will have higher pathogenicity than exotic isolates. This might be due to the difference in pathogenicity between the geographic region of the isolates and the insect host.

## Materials and methods

### Ethics statement

The red palm weevil different life stages were collected directly from the date palm orchard situated in Riyadh, Saudi Arabia. We declare that RPW stages were not collected from the public parks or protected areas. Moreover, it is not an endangered species in Saudi Arabia and no permits are needed to work on this species in the country.

### Red palm weevil colony

Different stages of RPW were collected from several date palm orchards in Riyadh. The colony was reared under 25 ± 2°C, 85 ± 5% relative humidity and 6:18 h L: D (photoperiod) using artificial diet. The artificial diet developed earlier by Al-Ayedh [25] was slightly changed to preserve texture and shelf-life by adding preservatives, antioxidants and agar. In the artificial diet, ground date palm petioles were used to provide natural flavor. The diet was prepared by adding a boiled mixture of potassium benzoate, sorbic acid, agar and distilled water to ground petiole, wheat flour, corn flour and ascorbic acid mixture after cooling to 60°C. The freshly hatched larvae were individually placed in plastic cups (d: 5 cm; h: 3 cm) and nourished with the artificial diet.

Existence of the hairs on adult weevil’s snout is used to identify the male and female. The presence of tiny hairs indicates that the weevil is male, whilst the absence of hairs indicates that it is female. The identified RPW females were transferred to a plastic container having sugar-soaked cotton to feed on and substrate for oviposition after mating. After 2 days, the eggs were collected, transferred to a Petri dish lined with water-soaked filter paper and left for hatching at 25°C. The larvae were transferred to an artificial diet in a plastic cup after hatching. The diet was changed at 1-week interval until the larvae reached the pupal stage. When the larvae were fully grown and stopped feeding, a 5-inch-long sugarcane set was provided to each larva for pupation. Newly emerged adults were collected from cocoons and transferred to the mating arena. After mating, the females were transferred to an egg-laying chamber. For the experiments, each of the RPW stage was of the similar age.

### Entomopathogenic fungi source

Different native isolates of *Beauveria bassiana* and *Metarhizium anisopliae* (originally from Al-Qatif governorate and Riyadh region) were obtained either from the Ministry of Agriculture or collected by the first author from Saudi Arabia. The exotic isolates collected from Kalimantan, Indonesia were used in this study. All isolates were assigned a code based on their origin (SA for Saudi Arabia), species (Bb for *B*. *bassiana*) and the codes were BbSA-1, BbSA-2 and BbSA-3. The *M*. *anisopliae* was coded as Ma and the isolate code was designated the code MaSA-1. Similarly, Indonesian isolates (IDN) of *B*. *bassiana* were coded as BbIDN-1 and of *M*. *anisopliae* as MaIDN-1, and MaIDN-2. Detailed information regarding the source of fungi are given in Table 1.

**Table 1:** Specific information about entomopathogenic fungi isolates used in the present study.

Isolate Name	Isolate Code	Insect Species/Order	Source of Isolation	Original	Coordinates
*B*. *bassiana*	BbSA-1	Red palm weevil/Coleopteran	Adult	Al Qatif, Saudi Arabia	N: 26.34437°; E: 43.69217°
*B*. *bassiana*	BbSA-2	Cotton leafworm/Lepidopteran	Larva	Al Qatif, Saudi Arabia	N: 24.41867°; E: 46.65408°
*B*. *bassiana*	BbSA-3	Red palm weevil/Coleopteran	Adult	Al Qatif, Saudi Arabia	N: 26.35231°; E: 43.71789°
*B*. *bassiana*	BbIDN-1	Corn earworm/Lepidopteran	Larva	Kalimantan, Indonesia	N: −0.02633°; E: 109.3425°
*M*. *anisopliae*	MaSA-1	Red palm weevil/Coleopteran	Adult	Riyadh, Saudi Arabia	N: 24.41867°; E: 46.65408°
*M*. *anisopliae*	MaIDN-1	Coconut rhinoceros beetle/Coleopteran	Adult	Kalimantan, Indonesia	N: −0.02633°; E: 109.3425°
*M*. *anisopliae*	MaIDN-2	Coconut leaf beetle/Coleopteran	Adult	Kalimantan, Indonesia	N: −0.03962°; E: 109.3128°

### Fungi isolation and purification

Fungi-infected RPW adults cadavers were sterilized and small part was dried on filter paper then transferred to potato dextrose agar (PDA) (Scharlau, Microbiology 01–483, Eur. Pharm) to grow at 25 ± 2°C and 85 ± 5% relative humidity [26]. A hyphen tip technique was used for fungi purification [27].

### Culture of fungi Isolates on potato dextrose agar medium

First purification of isolates was grown on PDA followed by screening of the isolates that germinated rapidly. The purification was performed 15 times through PDA medium to enhance the performance of the isolates. Conidia were produced from an isolated fungi cultivated on PDA plates for 14 days, after which each plate was supplemented with 10 ml sterile distilled water mixed with Triton-X (0.1%) and then harvested by scraping the inoculum [28]. The concentration of conidia was measured by hemocytometer (Improved Neubauer, Germany) and the final concentration was adjusted to 1 × 10^9^ conidia/ml.

### Bioassay procedures

Fungi isolates (1×10^9^ conidia/ml) were applied to different RPW stages by dipping method [15, 29, 30]. Based on the preliminary study, the concentration was selected sufficient for killing the RPW larvae. The mortality rates were calculated for statistical analysis in order to determine the relative efficacy of different isolates. Observations were taken daily until the individuals in the control were molted into next developmental stage and the average mortality time (days) was calculated.

### Pathogenicity tests on red palm weevil stages

The RPW eggs (1 day old) were treated with fungi isolates. The eggs were gently dipped in fungi solution (1×10^9^ conidia/ml) for 3 seconds and transferred to Petri dish (10 cm) having wet sterile filter paper. After bioassay, the eggs were kept in an incubator (Steridium, Australia) at 25 ± 2°C with 85 ± 5% relative humidity. The eggs were observed daily for 7 days to record the mortality of eggs and hatched larvae. There were three replicates and ten eggs in each replicate. Only sterilized distilled water was used in the control treatment.

The isolates were applied through dipping method for bioassay on larvae and pupae. The concentration of fungi isolates was 1×10^9^ conidia/ml. In case of larvae, different ages (3 and 35 days old) were used. Each larva was dipped in 20 ml fungi solution for 3 seconds [29], transferred to a new plastic cup having 5 g of artificial diet and covered with aerated lid. Similarly, wet filter paper was supplied for a pupa bioassay after individual dipping. The larvae and pupae were dipped in sterilized distilled water for control treatment. Samples undergoing each treatment were transferred to an incubator for 15–21 days. There were three replicates and five larvae in each replicate. The larvae and pupae were every 2^nd^ day. The dead larvae were shifted into sterile Petri dishes having moist filter paper and incubated at 25 ± 2°C with 85 ± 5% relative humidity to investigate fungal growth.

Pathogenicity of the isolates against adults was determined through dipping method. The adults were dipped into 20 ml fungi solution having concentration of 1×10^9^ conidia/ml for 3 seconds in a plastic container. Then, male and female adults (one pair) were transferred into new plastic cups were provided with half pieces of sugarcane (± 5 cm) and covered with an aerated lid. In this bioassay, 10-day-old adults were used. In the control, only distilled water was used. There were three replicates, each of which contained three pairs of adult males and females placed separately in a plastic cup. Samples undergoing each treatment were transferred to an incubator for 21 days. Following application, observations were performed every 2 days. The dead adults were incubated. The number of eggs/day produced by female weevils in each treatment were recorded.

### Experimental design

The bioassays were laid out according to completely randomized design.

### Statistical analysis

Non-hatching eggs, dead larvae, pupae, and adults were counted for percent mortality. The percent mortality was estimated using eggs that did not hatch and dead larvae, pupae and adults. After the incubation period, dead individuals of each RPW stage with unique symptoms such as fungi growth on their bodies; were considered infected by the fungi, while dead individuals without fungi infestation symptoms were excluded from the mortality percentage calculations. Fungi were considered as main effects and the dead RPW individuals as a response variable. The results were analyzed by one-way analysis of variance (ANOVA). The means were tested for significant differences using the least significant difference (LSD) test, with a threshold of P < 0.05 [31].

## Results

The results showed that all tested isolates were pathogenic against all RPW stages with different virulence. The highest mortality for all stages was recorded for MaSA-1, MaIDN-1 and BbSA-1 isolates. In addition, these isolates had high mortality rates on all RPW stages represented by faster killing, particularly on the egg and larval stages (3 days old).

### Egg mortality

The eggs were highly susceptible to all tested isolates compared to control treatment (Table 2). A significant difference was observed in egg mortality (F: 66.8; df: 7, 16; P: < 0.0001). In 1-day-old eggs, the average mortality of eggs and hatched larvae ranged between 90–100% for all tested isolates. There was a significant difference in mortality times of eggs caused by tested isolates (F: 141.5; df: 7, 16; P: < 0.0001) compared to control. All eggs were hatched in the control treatment.

**Table 2:** Mean mortality (% ± SE) of red palm weevil eggs treated with *Metarhizium anisopliae* and *Beauveria bassiana* isolates under laboratory conditions.

Treatments	Mortality (%)	Mortality time (days)
Control (water)	0 ± 0 b	0 ± 0 b
*Beauveria bassiana* (BbSA-1)	100 ± 0 a	4 ± 0 a
*Beauveria bassiana* (BbSA-2)	93.3 ± 6.6 a	4 ± 0 a
*Beauveria bassiana* (BbSA-3)	100 ± 0 a	4 ± 0 a
*Beauveria bassiana* (BbIDN-1)	90 ± 10 a	4 ± 0 a
*Metarhizium anisopliae* (MaSA-1)	100 ± 0 a	3.6 ± 0.3 a
*Metarhizium anisopliae* (MaIDN-1)	100 ± 0 a	4 ± 0 a
*Metarhizium anisopliae* (MaIDN-2)	100 ± 0 a	4 ± 0 a

Means followed by the same letter in the same column are not significantly different at α: 0.05.

A comparison of healthy (Fig 1A) and infected eggs (Fig 1B and 1C) is showing the effects of these fungi isolates.

**Fig 1:** Comparison of healthy and fungi-treated red palm weevil eggs. Healthy egg, exposed to distilled water (control) (A) and infected egg, exposed to fungi *Beauveria bassiana* (B) and *Metarhizium anisopliae* (C) (treated) (1 × 10^9^ conidia/ml) under laboratory condition.

### Larval mortality

Younger larvae (3 days old) were highly susceptible to all isolates compared to the older larvae (35 days old) (Table 3). The mortality rates of 3 and 35 days old larvae had significant differences (F: 22.46; df: 7, 16; P: < 0.0001; and F: 13.33; df: 7, 16; P: < 0.0001, respectively). The mortality rate ranged between 90%–100% in 3-day-old larvae with BbSA-1, BbIDN-1, MaSA-1 and MaIDN-1. The average larval mortality time was significantly different (F: 20.14; df: 7, 16; P: < 0.0001) than control. The highest mortality rate ranged between 86.6 to 93.3% in 35-day-old larvae with BbSA-1 and MaSA-1, respectively. The other isolates caused <73.3% mortality. In addition, there was a significant difference in mortality times of larvae caused (F: 83.31; df: 7, 16; P: < 0.0001) compared to the control. There was no mortality among the larvae in the control.

**Table 3:** Mean mortality (% ± SE) of 3 and 35 days old larvae of red palm weevil treated with *Metarhizium anisopliae* and *Beauveria bassiana* under laboratory conditions.

Treatments	Mortality (%)		Mortality time (days)	
	3-d-old larvae	35-d-old larvae	3-d-old larvae	35-d-old larvae
Control (water)	0 ± 0 c	0 ± 0 c	0 ± 0 c	0 ± 0 e
*B*. *bassiana* (BbSA-1)	100 ± 0 a	86.6 ± 6.6 a	7.6 ± 0.23 b	13.4 ± 0.53 cd
*B*. *bassiana* (BbSA-2)	86.6 ± 13.3 ab	53.3 ± 6.6 b	11.8 ± 0.61 a	15.8 ± 0.72 ab
*B*. *bassiana* (BbSA-3)	73.3 ± 6.6 b	53.3 ± 6.6 b	11.3 ± 0.66 a	15 ± 1.24 abc
*B*.*bassiana* (BbIDN-1)	100 ± 0 a	60 ± 11.5 b	8.4 ± 1.74 b	16.7 ± 0.15 a
*M*. *anisopliae* (MaSA-1)	100 ± 0 a	93.3 ± 6.6 a	6.9 ± 0.70 b	12 ± 0.26 cd
*M*. *anisopliae* (MaIDN-1)	93.3 ± 6.6 ab	73.3 ± 6.6 ab	7 ± 0.11 b	14.2 ± 0.26 d
*M*. *anisopliae* (MaIDN-2)	80 ± 11.5 ab	60 ± 11.5b	8 ± 0.86 b	15 ± 0.47 bc

Means followed by the same letter in the same column are not significant different at α: 0.05.

A comparison of healthy (Fig 2A) and infected larvae (Fig 2B, 2C, and 2D) exhibits clear effects of these fungi isolates.

**Fig 2:** Comparison of healthy and fungi treated red palm weevil larvae. Healthy larvae, (3 and 35 days old) exposed to distilled water (control) (A), early symptoms of infection (1 day after dead) by fungi (B), and infected larvae (3 and 35 days old), exposed to fungi *Beauveria bassiana* (C) and *Metarhizium anisopliae* (D) (treated) (1 × 10^9^ conidia/ml) under laboratory condition.

### Pupal mortality

There were significant differences in pupal mortality rate caused by tested isolates (F: 18.2; df: 7, 16; P: < 0.0001) (Table 4). The highest mortality (73.3–80%) was noted for BbSA-1 and MaSA-1. The remaining isolates caused <66.6% mortality, while it as 6.6% in the control treatment. The mortality times of treated pupae and control were significantly different (F: 4.1; df: 7, 16; P: < 0.0088).

**Table 4:** Mean mortality (% ± SE) of pupae of red palm weevil treated with *Metarhizium anisopliae* and *Beauveria bassiana* under laboratory conditions at 25 ± 2°C and 85 ± 5% RH.

Treatments	Mortality (%)	Mortality time (days)
Control (water)	6.6 ± 6.6 c	2.6 ± 2.6 b
*Beauveria bassiana* (BbSA-1)	73.3 ± 6.6 ab	8 ± 0 a
*Beauveria bassiana* (BbSA-2)	60 ± 6.6 b	8.6 ± 0.3 a
*Beauveria bassiana* (BbSA-3)	66.6 ± 6.6 ab	8.3 ± 0 a
*Beauveria bassiana* (BbIDN-1)	66.6 ± 6.6 ab	8.3 ± 0.3 a
*Metarhizium anisopliae* (MaSA-1)	80 ± 0 a	7 ± 0.3 a
*Metarhizium anisopliae* (MaIDN-1)	66.6 ± 6.6 ab	8 ± 0 a
*Metarhizium anisopliae* (MaIDN-2)	60 ± 0 b	8 ± 0 a

Means followed by the same letter in the same column are not significant different at α: 0.05.

A comparison of healthy (Fig 3A) and infected pupae (Fig 3B and 3C) shows clear effects of these isolates on pupa.

**Fig 3:** Comparison of healthy and fungi treated red palm weevil pupae. Healthy pupae exposed to distilled water (control) (A) and infected pupae exposed to fungi *Beauveria bassiana* (B) and *Metarhizium anisopliae* (C) (treated) (1 × 10^9^ conidia/ml) under laboratory condition.

### Adult mortality

Two isolates were selected for adult mortality bioassays and both differed for mortality (F: 51.8; df: 2, 6; P: < 0.0002) (Table 5). The highest mortality (74.3%) was caused by MaSA-1. The mortality times of treated adults and control were significantly different (F: 702.3; df: 2, 6; P: < 0.0001). Egg productions was significantly different (F: 84; df: 2, 6; P: < 0.0001) between treated adults and control.

**Table 5:** Mean mortality (% ± SE) of adults of red palm weevil treated with *Metarhizium anisopliae* and *Beauveria bassiana* under laboratory conditions.

Treatments	Mortality (%)	Mortality time (days)	Number of eggs laid by RPW females/day
Control (water)	0 ± 0 b	0 ± 0 b	4.2 ± 0.1 a
*Beauveria bassiana* (BbSA-1)	61 ± 5.5 a	16.8 ± 0.6 a	3 ± 0.1 b
*Metarhizium anisopliae* (MaSA-1)	74.3 ± 7.7 a	15 ± 0 a	3 ± 0.1 b

Means followed by the same letter in the same column are not significant different at α: 0.05.

A comparison of healthy (Fig 4A) and infected adults (Fig 4B and 4C) exhibits clear effects of these fungi isolates.

**Fig 4:** Comparison of healthy and fungi-treated red palm weevil adults. Healthy adults exposed to distilled water (control) (A), and infected adults, exposed to fungi *Beauveria bassiana* (B) and *Metarhizium anisopliae* (C).

In this study, MaSA-1 caused high mortality (100%, 100%, 93.3%, 86.6% and 74.3% in eggs, larvae, pupae and adults, respectively) compared to the remaining isolates and control. The BbSA-1 isolate caused 100%, 100%, 86.6%, 73.3% and 61% mortality in eggs, larvae, pupae and adults, respectively. The MaSA-1 isolate seemed very promising and effective against different RPW life stages.

## Discussion

Results show that high concentrations of fungi isolates caused higher mortality rates, as more conidia give a better chance of successful infection. Increased *B*. *bassiana* and *M*. *anisopliae* concentrations at 1 × 10^7^–1 × 10^9^ conidia/ml resulted in high mortality rates in different RPW life stages [14, 32, 33]. The *B*. *bassiana* isolated from infected RPW pupae have the potential to infect RPW stages at concentrations of 1 × 10^7^ to 1 × 10^9^ conidia/ml [15]. In addition, *B*. *bassiana* and *M*. *anisopliae* isolates were tested under laboratory conditions at different concentrations (1 × 10^3^ to 1 × 10^5^ conidia/ml) which caused 100% larval mortality in RPW within 9 days at a high concentration [34].

The present study confirmed the insecticidal activities of native and exotic isolates against different life stages of RPW under laboratory conditions. In our study, 90–100% egg mortality was observed with all isolates. The *M*. *anisopliae* isolates had high pathogenicity on eggs. This is supported by earlier studies showing that *M*. *anisopliae* caused high mortality rates (83%) in RPW eggs [14]. Similarly, *B*. *bassiana* and *M*. *anisopliae* caused a reduction of egg hatchability above 80% in peach borer (coleopteran) upon immersion with 1 × 10^8^ conidia/ml [35].

In our study, local isolates showed greater pathogenicity on the youngest and oldest larvae, in contrast to exotic ones. These results have been confirmed with the use of *B*. *bassiana* and *M*. *anisopliae* isolates with 1 × 10^10^ conidia/ml concentrations, which caused 83–100% mortality in larvae aged three to seven days. Local fungi isolates were more promising than commercial ones [36]. This result was consistent with other studies in which *B*. *bassiana* and *M*. *anisopliae* isolates showed increased mortality rates for early-instar RPW larvae [37]. In addition, other results confirmed that differently aged first and third instar larvae of rhinoceros beetle (*Oryctes rhinoceros*) showed different mortality rates [38]. Likewise, local fungi isolates isolated from adult RPW observed 90–100% mortality under laboratory conditions [36]. In our study, *M*. *anisopliae* caused 93.3–100% larval mortality after 6.9 to 12 days of inoculation at a concentration 1×10^9^ conidia/ml through dipping method. However, 60% of RPW larvae were killed by *M*. *anisopliae* ZJ-1 at a concentration 1×10^6^ within 10 days, while 100% was achieved at a concentration of 1×10^8^ within 8 days, when the fungi contacted the larvae by spraying [32].

In our study, RPW pupal mortality rates varied for all tested isolates. One of the local *M*. *anisopliae* isolates showed the highest pathogenicity against the pupae. This was supported by other studies indicating higher virulence of the *Metarhizium* genus on pine weevil pupae compared to the *Beauveria* genus [39].

In our study, local *B*. *bassiana* and *M*. *anisopliae* isolates still had good potential to kill RPW adults compared to exotic isolates. In addition, *B*. *bassiana* and *M*. *anisopliae* caused 100% mortality at a concentration of 1 ×10^9^ conidial/ml; thus, have potential to control coleopteran beetles such as adult bark beets [40]. However, *M*. *anisopliae* was reported to be the most virulent isolate, causing 100% mortality of RPW adults in contrast to *B*. *bassiana* and *Paecilomyces sp*., within 12 days at a concentration of 5×10^7^ for 120 seconds [33]. These published reports support our findings showing that *M*. *anisopliae* (MaSA-1) was the most virulent isolate. In this study, the adult RPW mortality rates were 61% and 74.3% for BbSA-1 and MaSA-1 isolates, respectively. Similarly, egg production from treated females was lower than control ones, but no disease transmission or infection of eggs or hatched larvae occurred. However, egg production was reduced by 27.4% in treated adults compared to the control. The mortality rate of RPW adult was 32.8% and 70% reductions in offspring of untreated females and contaminated males; however, there was a 60% risk of disease transmission to healthy RPW adults [15]. Our study confirmed the findings of other studies, with RPW adults infected by *M*. *anisopliae* showing symptoms, including the absence of darkening of the body after death and a high level of sporulation [33]. However, our study also showed high sporulation due to *M*. *anisopliae* in dead RPW eggs, larvae, pupae and adults.

Variation in the host range, pathogenicity and virulence of different fungi strains has been reported earlier [29, 41]. Generally, fungi have specific insect hosts; for example, *M*. *acridum* specifically kills grasshoppers [42]. However, *B*. *bassiana* and *M*. *anisopliae* have wide host ranges [41]. In our study, several isolates were associated with different responses regarding the pathogenicity against RPW stages, which might be due to different effects of geographical factors between the local and exotic isolates. This result explained that genetic variability between different *B*. *bassiana* isolates was investigated using inter-microsatellite (ISSR) with 80% polymorphism from different geographical locations with different pathogenicity [43].

Fungi isolates of *M*. *anisopliae* var. *acridum* isolated from lepidopteran larvae and adults were reported to be more effective against RPW larvae than *B*. *bassiana* isolated from coleopteran beetles [34]. Similarly, *M*. *anisopliae* has been shown to have a higher mortality rate against different RPW life stages than *B*. *bassiana* [14]. In comparison with other isolates, *B*. *bassiana* exhibits strong virulence toward larvae and adults of RPW [29]. However, the mortality times for local and exotic fungi isolates also varied in our study. These results were confirmed by other studies in which the mortality time difference for *B*. *bassiana*-infected RPW stages included 4 days, 4 days and 21 days for eggs, fourth-instar larvae and adults, respectively [15]. In our study, *M*. *anisopliae* (MASA-1) showed that RPW stages have a higher mortality rate and we suggest that RPW ages as well as stages have played a significant role in the fungi isolates infection process.

## Conclusion

The present research findings proved that native fungi isolates have strong pathogenic activity against RPW under laboratory conditions. In future research, focus should be placed on using the most virulent fungi isolates under field conditions for RPW management. Based on the present study we are confident enough to recommend to use *Metarhizium anisopliae* isolate in the field applications since it has proved to be a promising isolate.
